The article "Epithelial–Myoepithelial Carcinoma of the Esophagus: A Case Report" was published in 2022. Journal: Front Surg.

# Epithelial–Myoepithelial Carcinoma of the Esophagus: A Case Report

**DOI:** 10.3389/fsurg.2022.942019

**Published:** 2022-07-06

**Authors:** Haohao Wu, Fangbiao Zhang, Jiahui Peng, Zhiju Wu, Xiangyan Zhang, Xingzhen Wu

**Affiliations:** ^1^ Department of Emergency, Zhejiang University, Lishui Hospital, Lishui Municipal Central Hospital, Lishui, China; ^2^ Department of Cardiothoracic Surgery, Zhejiang University, Lishui Hospital, Lishui Municipal Central Hospital, Lishui, China; ^3^ Department of Pathology, Zhejiang University, Lishui Hospital, Lishui Municipal Central Hospital, Lishui, China; ^4^ Department of Rehabilitation Medicine, Zhejiang University, Lishui Hospital, Lishui Municipal Central Hospital, Lishui, China

**Keywords:** epithelial, myoepithelial, carcinoma, esophagus, surgery

## Abstract

Epithelial–myoepithelial carcinoma (EMC) of the esophagus is a rare biphasic tumor with low malignant potential, which has not previously been reported in the published literature. The present study describes the case of an asymptomatic, 53-year-old male who presented with EMC in the esophagus during a gastroscopic examination. Esophageal computed tomography (CT) showed thickening of the wall of the lower esophagus with a thickness of about 0.7 cm, and an enhanced scan showed uneven enhancement of the thickened esophageal wall. Thoracoscopic esophagectomy was performed because the tumor was malignant. Histopathology revealed that the tumor was characterized by a biphasic architecture consisting of cuboidal ductal cells and myoepithelial cells. The patient’s postoperative recovery was eventful, an anastomotic fistula occurred, and the patient was discharged from the hospital after 84 days. One year postsurgery, the patient remained in good health, with no evidence of metastasis and recurrence.

## Introduction

Epithelial–myoepithelial carcinoma (EMC) is a rare malignant tumor comprising epithelial cells and myoepithelial cells, which was initially described by Donath in 1972 (1). Since its discovery, EMC has been identified in several locations, including the parotid gland, minor salivary glands (especially the palate), respiratory tract, maxillary sinus, larynx, lungs, and penile. Furthermore, the most common site is the parotid gland (2). Patients often do not exhibit obvious clinical symptoms in the early stage of an esophageal tumor. As the tumor grows, patients present with different symptoms that are dependent on tumor size and location, including progressive dysphagia, chest pain, and hoarseness. Due to the rarity and unproven malignant potential of esophageal EMC, the available treatment is still uncertain. According to previous reports, surgery remains the best treatment option for EMC at other sites. Here, we report a case of EMC of the esophagus in a 53-year-old male that was treated with thoracoscopic esophagectomy and review the previously reported cases.

The article "Epithelial–Myoepithelial Carcinoma of the Esophagus: A Case Report" was published in 2022. Journal: Front Surg.

## Case Presentation

A 53-year-old asymptomatic male presented to the Lishui Municipal Central Hospital (Lishui, China) with a mass discovered on gastroscopy due to a routine medical examination. He had a history of smoking 40 cigarettes per day for 30 years and no history of diabetes mellitus, hepatitis, hypertensive disease, and tuberculosis. Written informed consent was obtained from the patient for the publication of the present study. Gastroscopy revealed a mass in the lower esophagus with rigid tissue (Figure 1). Pathological examination indicated heterotrophic hyperplasia of epithelial cells and possible malignancy. Esophageal CT (Philips, Brilliance ICT CP 200063) showed thickening of the wall of the lower esophagus with a thickness of about 0.7 cm, and an enhanced scan showed uneven enhancement of the thickened esophageal wall. A preoperative diagnosis of esophageal cancer was considered due to the gastroscopic pathological examination and enhanced CT features. Other physical examinations, including lung functional examination, electrocardiogram, abdominal ultrasound, brain magnetic resonance imaging (MRI), and radionuclide bone imaging, were normal. The serum levels of the tumor markers (alpha fetal protein, carcinoma embryonic antigen, squamous cell carcinoma antigen, carbohydrate antigen (CA)72-4, CA199, CA125, and cytokeratin 19 fragment) were within normal limits. Due to the possibility that the mass was malignant, a thoracoscopic esophagectomy was performed under general anesthesia on May 31, 2021. Intraoperatively, the tumor was in the lower esophagus and the tissue was tough. The tumor measured 20 mm and was present along the esophageal wall. Pathological examination revealed the tumor was characterized by biphasic architecture consisting of cuboidal ductal cells and myoepithelial cells (Figure 2). On immunohistochemistry, the duct-forming epithelial cells were positive for cytokeratin 7 (Figure 3). The outer cells were positive for p40, p63 (Figure 4), and cytokeratin 5/6, suggesting a myoepithelial phenotype. The Ki-67 labeling index was about 20% (Figure 5). The patient's postoperative recovery was eventful, an anastomotic fistula occurred, and the patient was discharged from the hospital after 84 days. Due to the esophageal anastomotic fistula resulting in anastomotic local scar hyperplasia, the patient underwent esophageal dilation three times. One year postsurgery, the patient remained in good health, with no evidence of metastasis and recurrence.

The article "Epithelial–Myoepithelial Carcinoma of the Esophagus: A Case Report" was published in 2022. Journal: Front Surg.

**Figure 1:** Gastroscopy revealing a mass in the lower esophagus with rigid tissue.

**Figure 2:** Pathological examination revealing that the tumor was characterized by biphasic architecture consisting of cuboidal ductal cells (black arrow) and myoepithelial cells (red arrow) (200×).

**Figure 3:** On immunohistochemistry, the duct-forming epithelial cells were positive for cytokeratin 7 (200×).

**Figure 4:** Outer cells positive for p63, suggesting a myoepithelial phenotype (200×).

**Figure 5:** Ki-67 labeling index of about 20% (100×).

## Discussion

EMC is a rare biphasic tumor with low malignant potential that accounts for 1% of salivary gland tumors (3). The most common location is parotid, and a small proportion occurs in the submandibular gland and small salivary gland (4). In addition to the salivary glands, EMC rarely occurs in other parts of the body, including the lungs (2), palate (5), penis (6), and so on. Due to its varied histopathologic appearance, EMC was first reported by Donath in 1972 (1) and subsequently recognized as a distinct tumor type starting in 1991 (7) by the World Health Organization (WHO).

The symptoms may be similar to esophageal cancer. In the early stages of esophageal EMC, patients often do not exhibit clinical symptoms. In the late stages, patients present with progressive dysphagia, chest pain, and so on. Imaging examinations, including chest CT and barium esophagram, are used for assessing esophageal EMC. There are limited data on chest CT and barium esophagram imaging features of esophageal EMC. The available data show that esophageal EMCs are esophageal stenosis or thickening of the esophageal wall, but they are nonspecific. Gastroscopy is the most effective preoperative examination method. It can observe the shape and size of the tumor and take a biopsy to confirm the diagnosis.

The definitive diagnosis of EMC depends on the results of pathological examination and immunohistochemistry. EMC displays a typical histological biphasic comprising an epithelial cell component surrounded by clear cells of myoepithelial origin (2). On immunohistochemical staining, the outer myoepithelial cells reveal the expression of myoepithelial cell markers, including calponin, p63, smooth muscle actin, vimentin, h-caldesmon, muscle-specific actin, S100, and smooth muscle myosin (5). By contrast, the inner epithelial cells are negative for myoepithelial markers and demonstrate immunoexpression of epithelial cell markers such as cytokeratins, carcinoembryonic antigen (CEA), and epithelial membrane antigen (EMA) (5). In the present case, hematoxylin and eosin (H&E) staining of typical EMC reveals epithelial cells surrounded by myoepithelial cells. Furthermore, positive CK7 expression of epithelial cells and positive p63 expression of myoepithelial cells are important markers for the diagnosis of an EMC.

The article "Epithelial–Myoepithelial Carcinoma of the Esophagus: A Case Report" was published in 2022. Journal: Front Surg.

Due to the rarity and unproven malignant potential of these tumors, the definite treatment protocol is still unknown. According to previous reports, surgery remains the safe and effective treatment option for EMC of other sites in the body. Complete surgical excision of the tumor provides superior outcomes in terms of survival and recurrence rates. Due to the lack of sufficient reported cases, there is insufficient evidence for postoperative chemoradiotherapy. Mori (2) described the case of a 72-year-old male who was diagnosed with primary pulmonary EMC. The patient received a thoracoscopic left upper lobectomy and no adjuvant therapy. At the 4 years of follow-up, the patient with no metastasis and recurrence but rectal cancer was subsequently diagnosed and died quickly. Similarly, Nakashima (8) reported a case of EMC that occurred in the lung. The patient received a right pulmonary middle lobectomy along with hilar and mediastinal lymph node dissections. At the 36th month of follow-up, the patient is doing well without any sign of recurrence. Safiullah (6) reported a case of EMC that occurred in the penile. The patient received uncomplicated local wide excision and no antitumor therapy. The patient was asymptomatic 1 year after surgery. In our case, we performed surgical treatment based on our experience with esophageal cancer. At the 1 year of follow-up, the patient was asymptomatic.

## Conclusion

In conclusion, the present study described a rare case of esophageal EMC in a male patient. To the best of our knowledge, a case of EMC in the esophagus has never been reported to date. Identifying diagnosis and effective treatment remains a challenge. However, complete surgical excision is still considered the most effective treatment.

## Data Availability

The original contributions presented in the study are included in the article/Supplementary Material; further inquiries can be directed to the corresponding author/s.
